The article "Deep Learning-Based Image Segmentation of Cone-Beam Computed Tomography Images for Oral Lesion Detection" was published in 2021. Journal: J Healthc Eng.

# Deep Learning-Based Image Segmentation of Cone-Beam Computed Tomography Images for Oral Lesion Detection

**DOI:** 10.1155/2021/4603475

**Published:** 2021-09-21

**Authors:** Xueling Wang, Xianmin Meng, Shu Yan

**Affiliations:** ^1^Department of Stomatology, Aerospace Center Hospital, Beijing 100049, China; ^2^Department of Stomatology, PLA Strategic Support Force Characteristic Medical Center, Beijing 100101, China

## Abstract

This paper aimed to study the adoption of deep learning (DL) algorithm of oral lesions for segmentation of cone-beam computed tomography (CBCT) images. 90 patients with oral lesions were taken as research subjects, and they were grouped into blank, control, and experimental groups, whose images were treated by the manual segmentation method, threshold segmentation algorithm, and full convolutional neural network (FCNN) DL algorithm, respectively. Then, effects of different methods on oral lesion CBCT image recognition and segmentation were analyzed. The results showed that there was no substantial difference in the number of patients with different types of oral lesions among three groups (*P* > 0.05). The accuracy of lesion segmentation in the experimental group was as high as 98.3%, while those of the blank group and control group were 78.4% and 62.1%, respectively. The accuracy of segmentation of CBCT images in the blank group and control group was considerably inferior to the experimental group (*P* < 0.05). The segmentation effect on the lesion and the lesion model in the experimental group and control group was evidently superior to the blank group (*P* < 0.05). In short, the image segmentation accuracy of the FCNN DL method was better than the traditional manual segmentation and threshold segmentation algorithms. Applying the DL segmentation algorithm to CBCT images of oral lesions can accurately identify and segment the lesions.

## 1. Introduction

In recent years, with the development of computer technology and its popularity in various fields, medical institutions and other fields have been combined with computer technology, and computer-aided means are widely utilized. At present, computed tomography and magnetic resonance imaging (MRI) are widely adopted in the medical field [1]. CT is a type of X-ray computed tomography, in which different tissues absorb different amounts of X-rays. This technology can be applied to display the internal structure of the human body in the form of three-dimensional imaging, thus providing convenience and basis for clinical diagnosis and treatment of diseases and related research [2]. As a feedforward neural network, the CNN can effectively reduce the complexity of the feedback neural network, which can be utilized to identify some two-dimensional images with distorted and nondeformed forms such as displacement and scaling. The extensive application of DL in medical image classification, such as CNN, can provide convenience for researchers based on traditional research methods [3, 4]. CBCT is a cone-beam projection computer recombination tomography influence device. The X-ray generator surrounds the projection body with a low amount of radiation to make a circular digital projection [5, 6]. The projection data are two-dimensional, and a three-dimensional image will be obtained after reconstruction. Image segmentation is the main step and operation from image processing to image analysis. At present, the most commonly utilized segmentation methods are threshold-based, region-based, edge-based, and specific theory-based techniques [7, 8]. In addition, the artificial neural network recognition technology has begun to attract attention and is widely applied in image segmentation. The neural network has a large number of connections and is easy to introduce spatial information, which can better solve the problems such as uneven distribution and noise in image recognition [9].

The article "Deep Learning-Based Image Segmentation of Cone-Beam Computed Tomography Images for Oral Lesion Detection" was published in 2021. Journal: J Healthc Eng.

Oral lesions include apical periodontitis, alveolar abscess, pericoronitis, periodontitis, and jaw osteomyelitis. When the oral lesion is stimulated by the external environment, the pathogenic microorganisms and related products in the lesion will diffuse outward. Then, damage to other systems or tissues and organs is caused, such as rheumatoid arthritis, chronic glomerulonephritis, erythema multiforme, and purulent nephropathy, which will aggravate the condition. However, the application of DL segmentation algorithm to oral lesion CBCT images is relatively lacking, and it is imperative to conduct in-depth research to study its clinical application [10, 11].

In this work, patients with oral lesions treated in the hospital were selected and divided into three groups and then the manual segmentation method, threshold segmentation algorithm, and FCNN DL algorithm were adopted for comparative research. They were applied to oral lesion CBCT image recognition and segmentation, so as to analyze and discuss the influence of FCNN DL algorithm on oral lesion and its effect on CBCT image analysis.

## 2. Materials and Methods

### 2.1. Selection and Grouping of Research Subjects

90 patients who underwent oral lesion treatment in the hospital from September 2018 to September 2020 were selected as the research subjects, including 48 male patients and 42 female patients. Patients who voluntarily withdrew and transferred to the hospital were excluded. The included patients were randomly classified as three groups, blank group (manual segmentation method), control group (threshold segmentation algorithm), and experimental group (FCNN DL segmentation algorithm), with 30 cases in each group.

The article "Deep Learning-Based Image Segmentation of Cone-Beam Computed Tomography Images for Oral Lesion Detection" was published in 2021. Journal: J Healthc Eng.

Inclusion criteria were as follows: (i) patients aged between 40 and 60; (ii) patients with clear consciousness and who could cooperate with treatment and sample collection; (iii) patients diagnosed with oral lesions; (iv) patients with complete clinical data and information; (v) patients without a history of mental illness and emotional stability.

Exclusion criteria were as follows: (i) patients who withdrew and transferred for treatment due to personal reasons; (ii) patients with other serious diseases or infectious diseases; (iii) patients with severe oral lesions or patients who had undergone treatment for similar diseases; (iv) patients with diseases of other systems or organs; (v) patients who had not received cooperative treatment due to personal or other reasons.

### 2.2. CBCT Data Set and Indicators

CBCT data of selected experimental sample patients were collected, and 90 patients with oral lesion CBCT data containing the final pathological test report were screened and selected. The CBCT data set contained CBCT cross-sectional images of patients with various oral lesions such as jaw osteomyelitis, periapical periodontitis, periodontal abscess, and pericoronitis. The image contained the overall three-dimensional structure of each patient's oral cavity, and the entire data set contained multiple CBCT images. The images were marked according to the type of the corresponding patient's lesion, and the above image marking was based on the medical gold standard of pathology test report and was jointly marked by multiple professional medical staff. After the labeling was completed, the corresponding preprocessing of the image was carried out. The CBCT images with value less than 0 were screened and set to 0, and the CBCT images with value greater than 3000 were screened and set to 3000. Then, the resulting image was divided by 3000 and multiplied by 255 to convert it into unit 8 digital format, and the preprocessed image was saved in the JPG image format. Finally, the accuracy and sensitivity of its classification were taken as evaluation indicators. The function of the denoising method in the two-dimensional image is defined as equation (1), and the function of the denoising method in the CBCT data CNN is defined as equation (2) in the three-dimensional space.

(1) $$\begin{array}{c} A\left(x,y\right)=\frac{1}{2\pi \theta^{2}}a^{\left(x^{2}+y^{2}/2\theta^{2}\right)}, \end{array}$$

(2) $$\begin{array}{c} A\left(x,y,z\right)=\frac{1}{2\sqrt{2}\pi^{1.5}\theta^{3}}a^{\left(x^{2}+y^{2}+z^{2}/2\theta^{2}\right)}. \end{array}$$

*A* represents the weight of each pixel; *θ* is the Gaussian distribution standard deviation parameter; the value of *θ* is 1.5; *x* is the abscissa value of the current pixel relative to the center pixel; and *y* is the abscissa value of the current pixel relative to the center pixel.

The article "Deep Learning-Based Image Segmentation of Cone-Beam Computed Tomography Images for Oral Lesion Detection" was published in 2021. Journal: J Healthc Eng.

### 2.3. Three Different Segmentation Algorithms for CBCT Image Segmentation

Manual segmentation: manual image segmentation should be performed by doctors with rich clinical experience and over 10 years of experience in the evaluation of oral diseases. The doctor evaluated and analyzed oral lesions and utilized mimics14.11 software to sketch out the edge of lesions on the oral CBCT image by hand.

Threshold segmentation algorithm: the segmentation method referred to CBCT image segmentation by setting appropriate tissue threshold in advance. The threshold was set on the mimics14.11 software, and the threshold of the 3D oral image model was set. The HU value region was preliminarily selected and the tissues under this region were monitored in real time. The selected area was slightly adjusted by medical professionals with extensive clinical experience until the threshold was set to the segmentation edge.

FCNN DL segmentation algorithm: the CNN can identify the image through sliding window, selective search, and other methods. This algorithm can identify and judge whether the window is the target object. Its recognition is defined as the regression problem of the occurrence probability of each target in image segmentation. This method adopts FCNN DL based on CBCT image segmentation to perform image segmentation on oral lesion evaluation and utilizes average crossover ratio as the final indicator.

(3) $$\begin{array}{c} R=\frac{|M\cap N|}{|M\cup N|}. \end{array}$$

*R* represents the average cross-union ratio, *M*={(*i*, *j*)} represents the point set that satisfies *Y*_*i*,*j*_ = 1 in the image, and *N*={(*i*, *j*)} represents the point set that satisfies *Y*_*i*,*j*_ > 0.5 in the image. The learning algorithm flow is shown in Figure 1.

### 2.4. Evaluation Indicators

The oral lesions of blank, control, and experimental groups were segmented according to the corresponding algorithm. The traditional manual segmentation, threshold segmentation algorithm, and FCNN DL algorithm were compared regarding the oral lesion CBCT image recognition and segmentation performance. Moreover, the running time, segmentation volume and surface area, image segmentation accuracy, and effect on lesions and lesion model segmentation of three methods were analyzed. The performances of the three algorithms were compared through the above indicators, and their recognition rate and accuracy of oral lesion image segmentation were studied.

The article "Deep Learning-Based Image Segmentation of Cone-Beam Computed Tomography Images for Oral Lesion Detection" was published in 2021. Journal: J Healthc Eng.

### 2.5. Statistical Analysis

The data were processed via the SPSS19.0 version software. Measurement data were expressed as mean ± standard deviation, and count data were expressed as percentage. The *t* test was adopted to compare the segmentation volume and surface area, as well as running time of manual segmentation, threshold segmentation, and FCNN algorithm. Analysis of variance was utilized to compare the segmentation effect of lesions and lesion models. The difference was statistically significant at *P* < 0.05.

## 3. Results

### 3.1. Location and Type of Oral Lesions in Patients of the Three Groups

The 90 patients selected for the treatment of oral lesions were diagnosed in the experiment, and the location of the lesion was judged, as shown in Figure 2. The oral lesions of the three groups of patients were mainly periodontal, pulpal, periapical, and other chronic oral inflammations. The incidence of periodontal lesions was the highest, reaching 38%, followed by dental pulp and periapical infectious lesions, which was 29% and 17%, respectively.

The types of lesions were periodontal abscess, apical periodontitis, and jaw osteomyelitis. The types of oral lesions that occurred in the three groups of patients and the number of patients with each type of lesion are statistically shown in Figure 3. Three oral lesions of periodontal abscess, periapical periodontitis, and jaw osteomyelitis occurred in each group of patients, and there was no evident difference in the number of patients with different types of oral lesions in the three groups (*P* > 0.05).

### 3.2. Local Oral Lesion

Figure 4 is a partial view of the lesion in a patient with periodontal abscess. The gums at the lesion site were red and swollen, with protruding abscess formation accompanied by abscess flow and submaxillary lymph node enlargement.

Figure 5 is a partial view of the lesion in a patient with apical periodontitis. There were obvious inflammatory changes in the surrounding tissues and swelling of the surrounding tissues, apical cysts, discoloration of teeth, and hyperplasia of granulation tissue at the mouth of the apical mucosal fistula.

### 3.3. Local Oral Lesion by Different Algorithms

Figure 6 shows the CBCT image of a patient with periapical periodontitis obtained by the traditional segmentation algorithm. The lesion site showed continuous and complete low signal; obvious edema, abscess, and inflammatory reaction were observed at the lesion site; and the lesion edge segmentation was incomplete.

Figure 7 is a CBCT image of a patient with apical periodontitis obtained by the tissue threshold segmentation algorithm. The lesion site showed uneven high signal, and the surrounding tissue showed a flat oval low-signal shadow. There were obvious inflammatory changes in the lesion site, and the lesion edge segmentation was relatively complete and clear.

The article "Deep Learning-Based Image Segmentation of Cone-Beam Computed Tomography Images for Oral Lesion Detection" was published in 2021. Journal: J Healthc Eng.

Figure 8 is a CBCT image of a patient with periodontal abscess by FCNN DL segmentation. Obvious abscesses appeared around the lesions and manifested as relatively loose mid-to-low-signal shadows, the edges of the lesions were completely segmented, and the lesion location was accurately identified.

### 3.4. Contrast of Segmentation Time and Accuracy of Three Segmentation Algorithms

Figure 9 shows the accuracy comparison results of the traditional segmentation algorithm, the tissue threshold segmentation algorithm, and the FCNN DL segmentation algorithm for oral lesion CBCT image segmentation. The segmentation accuracy of lesions in the experimental group was relatively higher and reached 98.3%, while those of the blank and control group were 78.4% and 62.1%, respectively. In contrast to the blank group, the accuracy of segmentation of CBCT images in the control and experimental group was notably higher (*P* < 0.05) and the accuracy of segmentation in the experimental group was considerably higher than in the control group (*P* < 0.05).

Figure 10 shows the comparison results of three segmentation algorithms for oral lesion CBCT image segmentation. The segmentation time of the FCNN DL segmentation algorithm was 10.2 ± 1.4 min, and that of threshold segmentation algorithm was 16.3 ± 1.6 min. The segmentation time of CBCT images in control and experimental groups was evidently shorter than in the blank group (*P* < 0.05), and the segmentation time in the experimental group was shorter than in control group (*P* < 0.05).

### 3.5. Contrast of Lesion Volume and Surface Area Obtained by Three Segmentation Algorithms

Figure 11 shows the comparison results of the volume and surface area of the oral lesion CBCT image segmentation by three segmentation algorithms. No evident difference was seen between the blank and experimental group in terms of split surface area and volume (*P* > 0.05). The volume and surface area in the control group were considerably smaller than in the blank group (*P* < 0.05), and the split volume and surface area in the experimental group were remarkably larger than in the control group (*P* < 0.05).

### 3.6. Segmentation Effect Comparison

Figure 12 shows the comparison results of the segmentation effects of the three segmentation algorithms on oral lesions and oral lesion models. The threshold segmentation algorithm and the FCNN DL algorithm had favorable segmentation effects on the lesion and the lesion model. The segmentation effect on the lesion and the lesion model in the experimental and control group was obviously superior to that in the blank group (*P* < 0.05). There was no substantial difference in the segmentation effect on lesions and lesion models between the control and experimental group (*P* > 0.05).

The article "Deep Learning-Based Image Segmentation of Cone-Beam Computed Tomography Images for Oral Lesion Detection" was published in 2021. Journal: J Healthc Eng.

## 4. Discussion

With the application and popularization of CBCT and other three-dimensional medical imaging technologies in medical testing and treatment, as well as the improvement of human lifestyle, oral health has gradually attracted attention [12]. Stomatologists have begun to try to apply CBCT to the detection and treatment of oral lesions. Since the visualization of CBCT images and data provides important reference value for medical personnel to detect through image segmentation and analysis, the occurrence and development of diseases can be monitored intuitively [13, 14]. Early medical image research and learning algorithms often have large limitations and are not suitable for the diagnosis and treatment of all diseases. In addition, most of the research is on the human brain, chest, and abdominal organs. Therefore, it is necessary to conduct in-depth research on image analysis and algorithms and apply them to oral diseases [15, 16]. According to statistics, the rate of oral diseases in China is only 9∼10%, which also has a great impact on oral health. Oral diseases, however, can cause serious bacterial or viral diseases if they fail to receive prompt diagnosis and treatment. Systemic diseases will even appear, such as chronic pharyngitis, rheumatoid arthritis, coronary heart disease, and chronic nephritis [17, 18]. In addition, relevant studies have found that oral therapy, such as periodontitis, has a bidirectional relationship with diabetes mellitus, in that severe periodontitis can aggravate diabetes mellitus and that patients' glycemic control ability is obviously worse than that of normal people. On the contrary, diabetes can also cause periodontitis and the bacteremia of periodontitis is likely to induce myocardial infarction and coronary heart disease [19]. Therefore, it is necessary to pay close attention to oral evaluation.

In this work, patients with oral lesions were selected and classified into three groups and then the manual segmentation method, threshold segmentation algorithm, and FCNN DL algorithm were adopted for comparative study. They were applied to oral lesion CBCT image recognition and segmentation, to analyze and discuss the influence of FCNN DL algorithm on oral lesions and its effect on CT images. The results showed that the experimental group was remarkably better than the blank and control group in terms of running time and accuracy of lesion segmentation. The experimental group and control group were remarkably better than the blank group in terms of the segmentation effect of lesions and lesion models (*P* < 0.05). The results were consistent with the research results of Sharma et al. [20], showing that the image segmentation accuracy of the FCNN DL method was better than the traditional manual segmentation and threshold segmentation algorithms, for it reduced the running time. Applying the DL segmentation algorithm to oral lesion CBCT images can accurately identify and segment the lesions, providing convenience for treatment, which can be applied to clinical diagnosis and treatment.

The article "Deep Learning-Based Image Segmentation of Cone-Beam Computed Tomography Images for Oral Lesion Detection" was published in 2021. Journal: J Healthc Eng.

## 5. Conclusion

Based on the oral lesion CBCT images, the analysis and research on the FCNN DL segmentation algorithm were carried out. 90 patients were selected, and then, the DL algorithm was applied to their oral lesion CBCT images. The manual segmentation method, threshold segmentation algorithm, and FCNN DL algorithm were adopted to process images of patients in different groups for comparative study. It was found that the image segmentation effect accuracy of the FCNN DL was better than that of the traditional manual segmentation and threshold segmentation algorithms and the running time was notably reduced. The adoption of DL segmentation algorithm in oral lesion CBCT image segmentation can accurately identify and segment the lesions, which could provide convenience for treatment, and it was suitable to be applied in clinical diagnosis and treatment. However, the sample size selected in this study is small, which may have a certain impact on the experimental results, and the representativeness is low. Therefore, the sample size will be increased in subsequent experiments, and the influence of FCNN DL algorithm on oral lesion and CT image analysis will be further analyzed and discussed. In conclusion, this research provides data support and theoretical basis for the clinical diagnosis and treatment of oral lesions, as well as the adoption effect of FCNN DL segmentation algorithms on oral CBCT images.

## Figures and Tables

**Figure 1:** Schematic diagram of the DL segmentation algorithm flow.

**Figure 2:** Location of the patients' oral lesions.

**Figure 3:** Types of oral lesions and number of patients.

**Figure 4:** Periodontal abscess.

**Figure 5:** Periapical inflammation.

**Figure 6:** Traditional segmentation of the CBCT image of apical periodontitis.

**Figure 7:** CBCT image of apical periodontitis by the threshold segmentation algorithm.

**Figure 8:** CBCT image of the lesion by DL segmentation.

The article "Deep Learning-Based Image Segmentation of Cone-Beam Computed Tomography Images for Oral Lesion Detection" was published in 2021. Journal: J Healthc Eng.

**Figure 9:** Contrast of accuracy of three segmentation algorithms. Note: the symbols ^*∗*^ and ^#^ indicate that the difference was substantial, versus the blank group and control group, respectively (*P* < 0.05).

**Figure 10:** Contrast of running time of three segmentation algorithms. Note: the symbols ^*∗*^ and ^#^ indicate that the difference was substantial, versus the blank group and control group, respectively (*P* < 0.05).

**Figure 11:** Contrast of the surface area and volume of the three segmentation algorithms. Note: the symbols ^*∗*^ and ^#^ indicate that the difference was substantial, versus the blank group and control group, respectively (*P* < 0.05).

**Figure 12:** Comparison of the segmentation effects of three segmentation algorithms. Note: the symbols ^*∗*^ and ^#^ indicate that the difference was substantial, versus the blank group and control group, respectively (*P* < 0.05).

## Data Availability

The data used to support the findings of this study are available from the corresponding author upon request.
